# Multichannel CNN Model for Biomedical Entity Reorganization

This article has been retracted.

**DOI:** 10.1155/2022/5765629

**Published:** 2022-03-19

**Authors:** Ajay Kumar Singh, Ihtiram Raza Khan, Shakir Khan, Kumud Pant, Sandip Debnath, Shahajan Miah

**Affiliations:** ^1^Mody University of Science and Technology, India; ^2^Jamia Hamdard, Delhi, India; ^3^College of Computer and Information Sciences, Imam Mohammad Ibn Saud Islamic University (IMSIU), Riyadh, Saudi Arabia; ^4^Department of Biotechnology, Graphic Era Deemed to Be University, Dehradun, Uttarakhand, India; ^5^Department of Genetics and Plant Breeding, Palli Siksha Bhavana (Institute of Agriculture), Visva-Bharati University, Sriniketan, Birbhum, West Bengal, India; ^6^Department of EEE, Bangladesh University of Business and Technology (BUBT), Dhaka, Bangladesh

## Abstract

Biomedical researchers and biologists often search a large amount of literature to find the relationship between biological entities, such as drug-drug and compound-protein. With the proliferation of medical literature and the development of deep learning, the automatic extraction of biological entity interaction relationships from literature has shown great potential. The fundamental scope of this research is that the approach described in this research uses technologies like dynamic word vectors and multichannel convolution to learn a larger variety of relational expression semantics, allowing it to detect more entity connections. The extraction of biological entity relationships is the foundation for achieving intelligent medical care, which may increase the effectiveness of intelligent medical question answering and enhance the development of precision healthcare. In the past, deep learning methods have achieved specific results, but there are the following problems: the model uses static word vectors, which cannot distinguish polysemy; the weight of words is not considered, and the extraction effect of long sentences is poor; the integration of various models can improve the sample imbalance problem, the model is more complex. The purpose of this work is to create a global approach for eliminating different physical entity links, such that the model can effectively extract the interpretation of the expression relationship without having to develop characteristics manually. To this end, a deep multichannel CNN model (MC-CNN) based on the residual structure is proposed, generating dynamic word vectors through BERT (Bidirectional Encoder Representation from Transformers) to improve the accuracy of lexical semantic representation and uses multihead attention to capture the dependencies of long sentences and by designing the Ranking loss function to replace the multimodel ensemble to reduce the impact of sample imbalance. Tested on multiple datasets, the results show that the proposed method has good performance.

## 1. Introduction

With the development of the Internet, people have higher and higher requirements for information quality, and fields such as information extraction, information retrieval, machine translation, and knowledge graphs have become the focus of research. Among them, information extraction identifies and extracts specific factual information in a document and represents it in a structured and understandable form for users to query and use [1]. Named entity recognition (NER) is an essential task in information extraction. Its purpose is to identify the components representing named entities in the text. It is the basis for studying the semantic knowledge in the text. In addition, research in automatic question answering and opinion mining plays an important role [2]. In the early stage of the named entity recognition task, three main types of entities were identified. In extracting information, named entity recognition (NER) is an important task. Its goal is to find the components in the text that represent identified entities. It is the foundation for exploring into the text's semantic understanding. Furthermore, research into automatic question answering and opinion mining is critical. The message understanding conferences (MUC) stipulated that the three types of entities include named entities, time expressions, and quantity expressions. Driven by various evaluation conferences and natural language processing applications, the goals of designated entity recognition tasks continue to expand. The Automatic Content Extraction (ACE) project expands the geographical and institutional name entities, adding facility and geopolitical entities [3]. The Automatic Content Extraction (ACE) software is dedicated to extracting data using audiovisual inputs. The study attempt is limited to knowledge extraction from text, in contrast to simple text. The appropriate duty is to locate the specified element. It is a distinct problem, something that is more complex and requires more specific inferences in order to get a solution. The conference on natural language learning (CoNLL) adds other named entities to the MUC definition [4]. With the development of called entity recognition technology, the research on named entity recognition in specific fields has attracted the attention of researchers, and the research on named entity recognition in the area has gradually deepened, such as military field [5], agricultural field [6], and commodity field [7].

In biological cells, the regular operation of the entire organism is accomplished through the interaction between biological entities. As shown in Figure 1, in the process of metabolism, there are interactions of various biological entities, and problems in any one of them may lead to disorders of the body. The extraction of biological entity interaction has a wide range of applications in biomedical research. For example, protein-protein interactions play an essential role in many life processes that contribute to discovering drug targets for the treatment of disease [1]. Likewise, the adverse effects of drug-drug action impact people's health, with international medical organizations estimating that more than $4 billion is spent on the treatment of preventable adverse drug reactions every year [2]. Studying the interactions between biological entities is crucial for understanding the mechanisms of life and for pharmaceutical research and development. A better understanding of the interactions between proteins and small molecules is essential for a better understanding of molecular and cellular activities such as metabolism and signaling. Although information about such interactions is widely available across a variety of databases and literatures. As a result, gene encoding proteins that interact directly with various heavy metals or metalloids that have emerged as real hazards to the food chain through crops can be employed to breed novel genotypes with reduced levels of heavy metals or metalloids in the plant products. Those genes can be used to locate and construct gene-based molecular markers, and they may be targeted for further research purposes. [8].

Today, life science researchers routinely publish and disseminate research results into the scientific literature. At the same time, they frequently search the literature for domain-relevant information. The current volume of biomedical literature is enormous, and the growth rate far exceeds that of other fields of science. A large amount of biomedical knowledge exist in a large amount of literature in an unstructured form. It is not easy to retrieve and extract information from the literature manually. For example, the MEDLINE biomedical literature database established by the U.S. National Library of Medicine has collected 5,639 publications from 1950 to the present, with a total of more than 26 million literature records, and the current annual increase of 300,000 to 350,000 literature [9]. To effectively acquire relevant knowledge from the massive biomedical literature is a serious challenge faced by scholars in the biomedical field. With the development of text mining technology, the interaction relationship between biological entities can be automatically extracted from massive biomedical literature to facilitate life science researchers to obtain information and assist their research work, which will have a wide range of applications in life science research.

At present, with the development of deep learning, many works use deep methods to extract biological entity relationships, while the current position based on deep learning methods is still in its infancy. The Deep learning algorithms and an artificial neural network as classifiers were used to successfully identify identified things in digital medical data. Prior knowledge also plays a bigger role in boosting named entity identification tasks like knowledge graphs. The high efficiency of deep learning algorithm in named entity identification tasks, this study investigates and offers a strategy for mining and utilizing the most recent characteristics in plant attribute text. Most of the work still relies on domain experience to manually design features, combine the handcrafted elements with word vectors, and extract biological entity relationships through shallow models such as traditional CNN or LSTM. Since most of these features are designed on a limited training set, other datasets may not apply. In addition, some works improve prediction performance by fusing multiple shallow models, but this approach makes the model large and complex. Therefore, the purpose of this paper is to design a universal deep model, learn the semantics of expressing relationships through the model itself, and then extract various biological entity relationships. The method in this paper does not design additional features manually. Still, it only uses dynamic word vectors and position vectors as input, which enhances the robustness of the model, assigns vocabulary weights through the attention mechanism and uses residual units to form a deep multichannel CNN model. The model learns the characteristics of expressing relationships, and finally, through experiments, the method's effectiveness in this paper for the task of biological entity relationship extraction is verified.

The sequence labeling method assumes that for each word in the text (usually a word in Chinese), there are several candidate category labels, and the machine learning model is used to serialize and automatically label each word in the text. Typical machine learning models include the hidden Markov model [10] (hidden Markov model, HMM), support vector machine [11] (SVM), maximum entropy [2] (ME), and CRF (conditional random fields) [1]. The Hidden Markov Model plays an important role in the following fields, it offers a theoretical framework for creating comprehensive systems just by sketching an image. Gene finding, feature searches, related sequence recognition, and regulation site analysis are just a few of the tools that use them. It is a statistically stochastic model wherein the represented entity is believed to be a stochastic process (or “secret”) with unknowable (“secret”) state. With the development of deep learning technology, especially the emergence of the method of using word vectors to represent words, named entity recognition has brought a strong development impetus. Peng et al. drew on the good performance of LSTM (long and short-term memory) in automatic word segmentation. They proposed a model combining LSTM and CRF, which improved the *F* value by 5% compared with the previous method [12]. Lample et al. proposed two neural network models based on BiLSTM-CRF (bidirectional long short-term memory CRF) and conversion method, obtained features from labeled and unlabeled corpus simultaneously, and obtained comparable results in four languages. Literature [13] used deep learning technology and a convolutional neural network as a classifier to identify named entities in electronic medical records and achieved good results. In addition, prior knowledge has a better role in promoting named entity recognition tasks, such as knowledge graphs. Literature [14] used the open-source named entity system DBpedia Spotlight to optimize the named entity recognition task [3]. Based on the original system, the Chinese-related knowledge expands the candidate set incrementally. The point mutual information rate method is used in the feature selection of the entity context. Finally, the secondary disambiguation method based on the topic vector improves the annotation accuracy. Given the good performance of deep learning technology in named entity recognition tasks, this paper studies how to mine and utilize the latest features in plant attribute text and proposes a method. The method makes full use of the BiLSTM model to obtain the context and timing information of the plant attribute text. It uses the (convolution neural network) model to learn the latest features of the plant attribute text and then optimizes the CRF model to obtain the final sequence annotation results. The main contributions of this paper are as follows: propose named entity recognition based on BiLSTM, CNN, and CRF; study the adaptability of different models in the task of named entity recognition in plant attribute text.

## 2. Related Work

Extracting biological entity relationships through text mining has always been the focus of researchers. For example, in 1988, Swanson et al. [4] discovered the medical relationship between magnesium deficiency and migraine through literature mining. More and more researchers and organizations are involved in this work, such as the well-known text mining organization, Bio Creative (http://www.biocreative.org/), which organizes competitions on biomedical literature mining every year, actively promoting the development of research in this field. There are four main research methods for extracting biological entity interaction: entity word cooccurrence, pattern matching, machine learning, and deep learning methods. The cooccurrence frequency of entity words is often used to determine a relationship between entities. The online application STITCH developed in [5] is an example. But this method cannot provide the type and proof of the relationship. Pattern matching methods, such as the literature [6], use the maximum frequent sequence idea to automatically summarize the rules in the text and then mine the entity relationship. This method achieves high accuracy, but it is not easy to design a comprehensive model.

Moreover, the effect is closely related to the constructed features using machine learning methods. References [7, 15] use a two-stage approach to extract drug-drug relationships. First, by designing rich semantic features, determine whether there is a relationship between entities and then further classify the relationship, which is cumbersome. Recently, deep learning methods have developed rapidly, and the literature [16] proposed syntactic CNN, which uses syntactic word embedding to improve the model's performance. Reference [1] used the voting method to identify compound-protein relationships in the literature by combining models such as LSTM and CNN. However, the traditional techniques based on entity word cooccurrence and pattern matching cannot meet the current relationship extraction on the large-scale corpus. To capture relevant spatial patterns of diverse variables and integrate them to predict the yield response to fertilizer and seed rate control, a convolutional neural network (CNN) was utilized [17]. For the detection of *Aphis gossypii* glover infection in cotton leaves using hyperspectral Imaging, a multidimensional convolutional neural network (CNN) and a visualization method were integrated [18].

Complex algorithms and tools are required to handle raw data, ensure data quality, identify peptides and proteins, detect posttranslational modifications (PTMs), and perform further studies thereafter. In several elements of proteomics data processing, machine learning approaches have been widely adopted because of these computational needs [19–21, and]. Deep learning, a branch of machine learning, has previously been used to analyze gene expression and DNA and protein sequence data, and a wide range of biological data. Therefore, the use of deep learning in biomedicine, clinical diagnostics, bioinformatics, and genomics has thus been demonstrated [22]. The method based on machine learning needs to design a large number of professional features and train multiple classifiers for multiclassification problems, and the model is more complex [30]. At present, there is still a lot of room for improvement in the method using deep learning. These deep learning models use static word vectors and cannot generate corresponding word vectors for new and combined words. In addition, since the imbalance of positive and negative samples in the corpus affects the model's performance, previous methods usually use a model combination or filter samples to ensure sample balance [16, 23]. Still, filtering samples requires solid professional knowledge to design filtering rules, which the process is cumbersome and reduces the generalization of the model. Therefore, this paper proposes the MC-CNN model, which uses BERT [24] to generate dynamic word vectors. The same word in different sentences can generate other vector representations according to the context, overcoming the shortcomings of static word vectors.

Furthermore, to improve the extraction ability of long sentences, an attention mechanism is designed to enable the model to learn the internal dependency features of sentences. In addition, on the problem of sample imbalance, to maintain the original distribution of data, reduce manual intervention, and reduce costs, this paper does not filter negative samples but designs a loss function to minimise the impact of sample imbalance. Finally, the experimental verification shows that the proposed model has a good effect.

## 3. Problem Definition

The extraction of biological entity interaction refers to finding out the interaction information between arbitrary entities (such as proteins and drugs) in free text. Most of the current research is to extract sentence-level binary entity-relationship details, that is, to remove the role relationship between any two entities in a sentence. The field generally abstracts the task of relation extraction as a classification problem. First, some relationship categories are predefined by experts. When performing relationship extraction, it is necessary to design a method to identify which type the interaction between any two entities belongs to [3].

For example, in the compound-protein relationship extraction of Figure 2, the sentence “We conclude that erg3 can be blocked by sertindole and pimozide” contains three biological entities, which can be combined to form three entity pairs by pairwise combination. Researchers need to design methods to identify the relationship between these entity pairs, such as <erg3, sertindole> and < erg3, pimozide> relationship is “INHIBITOR” class. However, there is no relationship between <sertindole, pimozide>. This situation is usually classified as a specific category “OTHER” in multiclassification.

## 4. Methods and Models

### 4.1. Method Overview

The method in this paper is shown in Figure 3. First, the corpus is divided into a training set, validation set, and test set and preprocessed; then, BERT is used to generate dynamic word vectors; then, the attention mechanism is used to calculate the degree of correlation between words and learn the weight of words for further extraction through residual layer high-level semantic features; then, use multi-channel CNN to understand the semantics of expressing relationships and finally output the results predicted by the model through the prediction layer.

### 4.2. Input Data Representation

The input studied in this paper is text data, which needs to be converted into mathematical language when modeling. The commonly used method uses the distributed representation of vocabulary (also known as word embedding, word vector). Low-dimensional real-valued vectors represent the words in the input sentence, and then, the penalty is converted into a matrix. Word embeddings are learned from large-scale corpora, combining words with similar meanings. In the past, the word embeddings obtained by Word2Vec [2] were fixed, which could not solve the problem of word ambiguity. For example, “Bank” means both “bank” and “riverbank”. Therefore, BRET generates dynamic word embedding, which obtains a language model by modeling a large-scale corpus. When faced with a specific task, it can create word embeddings on the fly based on the input. The word embedding at this time combines the input context information, and different word embeddings will be generated for the same word in different scenarios, which solves the problem of polysemy. And for new words and compound words, BERT splits them into a combination of multiple short words, which completely avoids the situation that new words cannot find corresponding word embeddings. According to the assumption that words closer to the entity contribute more to the relationship, this paper adds relative position information to each word based on word embedding. In the example shown in Figure 2, the distances of “blocked” close to “erg3” and “sertindole” are 3 and −2, respectively.

### 4.3. Multihead Attention Mechanism

The previous models can only perform sequential calculations when processing sequence information, and it is challenging to capture long sentence-dependent information, so the extraction effect is not good. However, attention mechanism (attention) can solve this problem. The attention in this paper was proposed by Vaswani et al. [14]. It uses the inner vector product to represent the degree of correlation between two words, eliminating the influence of the distance between words and is no longer limited by sentences.

Multihead attention is a variant of the above attention. It splits the input into multiple parts, repeats the above calculation, and finally merges the results. The information of the multihead attention in this paper is the BERT-converted matrix of each sample, denoted as matrix *X*. The calculation process is shown in Figure 4. First, the input matrix *X* is subjected to three different linear transformations. The obtained query *Q* and key-value pairs *K* and *V* are divided into several parts. Then, each copy of *Q* and *K* is subjected to matrix multiplication, then scaled by dk times (dk is the latitude of the word embedding), and normalized by the softmax function to obtain the weight value, which is expressed as the degree of correlation between words. The weights and the corresponding *V* weights are then summed and combined. Finally, the combined output is linearly transformed to obtain the calculation result of the multihead attention. In this way, the split-merge calculation can get more information of the sample subspace and be executed in parallel during the calculation process, improving operation efficiency.

### 4.4. Multichannel Convolution Neural Networks

In image recognition, using multiple channels to provide information in different subspaces can improve the recognition ability of the model. Drawing on this point of view, this paper proposes a multichannel convolutional neural network to extract biological entity relationships. Many studies have shown that a deeper network can learn richer knowledge. Still, the deepening of the network will also lead to the problem of gradient disappearance and challenging training, and the introduction of residual units can avoid the above issues. To this end, the semantic information of the subspace is learned through the residual team to increase the input channels. As shown in Figure 5, the multichannel input is formed by stacking the output of the attention mechanism and the subspace semantic matrix generated by the residual unit, and each channel has semantic information of different granularity. Firstly, the sliding window operation is simulated according to the multichannel convolution and the feature ci of the phrase in window *i* is obtained. Then, use the maximum pooling to extract the feature words *p* that can express the relationship. Among them, Vk is the input of the kth channel, *C* is the number of channels, *W* is the convolution kernel parameter, *h* is the window size, *b* is the bias, *f* is the activation function, and *L* is the number of windows generated when the convolution kernel slides. The inclusion of residual units can alleviate the foregoing concerns by preventing gradient disappearance and challenging training as the network is deepened. To this purpose, the residual team learns the subspace's contextual features in order to enhance the input channels. The inter input is created by layering the focus mechanism's output and the residual unit's subspace semantic matrix, and each channel contains semantic information of varying granularity.

### 4.5. Prediction Layer

The prediction layer needs to calculate the probability corresponding to each relationship category and then use the class with the highest probability as the prediction result of the sample. As in Equation (1), using *m* different convolution kernels in a multichannel convolutional neural network will generate *m* different outputs. The number of related categories (denoted as *n*) is not equal to the number of convolution kernels, so the transformation operation shown in Equation (2) is required to transform them-dimensional vector *z* into an *n*-dimensional vector and then normalize it through the softmax function Transform to get the output *o*, where *W*_out_ is the transformation matrix, and each dimension of o = [o1, o2, ⋯, on] is a natural number in [0, 1], representing the probability corresponding to each relation category.

(1) $$\begin{array}{c} z=\left[p_{1},p_{2},\cdots ..p_{n}\right], \end{array}$$

(2) $$\begin{array}{c} o=\text{softmax }\left(W_{\text{out}}\;z\right) \end{array}$$

### 4.6. Loss Function

In the preprocessing stage, the entities of the same sentence are combined in pairs, which will result in a large number of entity pairs with no relationship, resulting in an imbalance of positive and negative samples. To this end, this paper adopts the Ranking-based loss function [25] as in Eq. (1), which does not train negative samples as a new category “OTHER” but adjusts the gradient update of negative samples by changing the edge factor. In the training process, when the model predicts a positive label as a negative label, the calculated gradient will be penalized so that the parameter update range is extensive, improving the severe imbalance between positive and negative samples. The loss function is calculated as follows:

(3) $$\begin{array}{c} L_{\mathrm{rank}}=\text{In}\left(1+\exp\left(\gamma \left(m^{+}-s_{y}\right)\right)\right.+\text{In}\left(1+\exp\left(\gamma \left(m^{-}-s_{c}\right)\right)\right., \end{array}$$

where *γ* is a scaling factor, and *m*^+^ and *m*^−^ are edge factors used to adjust the gradient update of positive and negative samples. *S* is the model prediction function, *y* is the actual label of the input sample, and *c* is the negative label with the highest score at the time of prediction. The training model phase set *γ* to 2.5, and *m*^+^ and *m*^−^ to be 3 and 0.5, respectively. In addition, L2 regularization is added to this loss function to speed up model training and improve generalization.

## 5. Experimental Results and Analysis

### 5.1. Dataset Description

To test the effect of the method in this paper, two commonly used biological entity-relationship datasets shown in Table 1 are selected. The DDI dataset is provided by the DDI Extraction 2013 challenge, which annotates five classes of relationships between drugs and drugs. Its data comes from two corpora, Pub-Med, and Drug-Bank. The former is a medical literature database, and the latter is a medicinal chemistry repository. The ChemProt dataset is provided by the BioCreative organization, which annotates ten types of relationships between compounds and proteins. Still, only five common relationships are officially evaluated, and the data are all derived from the Pub-Med literature database. There are significantly more negative samples than positive samples in these two datasets. Among them, the ratio of positive and negative examples in the DDI dataset is about 1 : 4.6, and the percentage of positive and negative samples in the ChemProt dataset is about 1 : 2.1, so it is necessary to train the model. First, consider the problems caused by sample imbalance.

### 5.2. Evaluation Metrics

The metrics commonly used to evaluate models in this field are precision *P*, recall *R*, and *F* values, which are defined as follows:

(4) $$\begin{array}{c} \text{Precision}\left(p\right)=\frac{\text{true Positive}\left(\text{tp}\right)}{\text{True Positive}\left(\text{tp}\right)+\text{false Postive}\left(\text{fp}\right)},\\ \text{Recall}\left(R\right)=\frac{\text{true Postive}\left(\text{tp}\right)}{\text{True positive}\left(\text{tp}\right)+\text{False negative}\left(\text{fn}\right)},\\ \text{F}1=\frac{2\text{PR}}{\text{P}+\text{R}}, \end{array}$$

where TP represents the number of positive samples predicted as positive classes, FP represents the number of negative models expected as positive classes, and FN represents the number of positive samples indicated as negative classes. Generally, the precision rate and the recall rate will restrict each other, so the *F* value is often used to measure the system's overall performance.

### 5.3. Analysis of Results

The model proposed in this paper is implemented using the open-source deep learning framework TensorFlow. Most of the structure of the model is a convolution neural network, with a significant degree of parallelism, and the use of GPU to accelerate the calculation can significantly reduce the training time.

Since some models are only evaluated on specific datasets, the analysis and comparison are performed on the two datasets separately. First, the proposed model is trained on the two datasets and then tested on the test set to calculate the corresponding evaluation indicators. Finally, the model's performance in this paper and the existing model are compared and analyzed. To ensure the rigour of the results, an average of 5 results was taken as the final result during the test. The evaluation results of other models are all from their original texts. Shown in Table 2 are the evaluation results on both datasets of the proposed methods in this paper.

As shown in Table 3 and Figure 6, the evaluation results on the DDI dataset show that the method proposed in this paper is comparable to other methods. SCNN [16] introduced syntactic information into the model by analyzing sentence structure and training syntactic word vectors. This approach has achieved some results, but some errors are generated when parsing the sentence structure, which will lead to the accumulation of model errors. Joint AB-LSTM [23] is composed of two LSTM-based submodels. The accuracy and *F* value of the model achieve the best results, indicating that the combination of models can reduce the error rate of relationship recognition. Still, the paper points out the prediction error. The proportion of long sentences is more significant in the samples, indicating that the model has a limited effect on long sentence extraction.

In contrast, the *F* value of the method in this paper is 0.9% different from the model with the best effect, but the model in this paper does not improve the impact through model fusion, so it is comparable. Further analysis found that the sample sentences from DrugBank in the DDI dataset are shorter, while the sample sentences from Pub-Med are longer. The attention mechanism proposed in this paper significantly improves the extraction effect of long sentences.

In contrast, the improvement of the extraction effect of short sentences is not apparent, which may be the main reason why this model fails to obtain the highest *F* value. The model in this paper has the highest recall rate, 2.2% higher than the best model, indicating that the method in this paper can identify more biological entity relationships, which proves the effectiveness of the way in the task of extracting drug-drug relationships.

The test results on the CHEMPROT dataset are shown in Table 4 and Figure 7. The Transfer Model [11] adopts the transfer learning method to initialize the model through the network parameters of related tasks so that the *F* value reaches 61.5%. The Ensemble Model [16] includes three independent models of SVM, CNN, and Bi-LSTMs, adds additional features to construct manually, and then obtains the highest accuracy through voting. Still, the model is relatively complex and challenging to transfer to others. GA-BGRU [12] uses bidirectional GRU units to extract semantic sentence features and the Swish activation function to improve the model effect.

In contrast, the method in this paper does not use a model ensemble. Still, it achieves the best results in both recall and *F* value through multichannel convolution operations, where the *F* value is 5.1% higher than the best method. Compared with the DDI dataset, there are more long sentences in the CHEMPROT dataset, and the overall effect is improved more obviously through the attention mechanism. This shows that the method in this paper can also well extract the relationship between compound and protein.

All in all, the model proposed in this paper performs well on the above two biological datasets, with the highest recall rates, as shown in Figure 8. The main reason is that the method in this paper learns a wider range of relational expression semantics through mechanisms such as dynamic word vectors and multichannel convolution, thereby identifying more entity relations. Furthermore, the multichannel CNN model proposed in this paper can significantly improve the recall rate. Experiments found that the recall rate has a special relationship with the number of multichannels. When the number of channels is set from 1 to 4, the recall rate improves significantly. The accuracy of the current model in this study and that of the existing model in comparison is examined. During the test, an average of five outcomes was used as the final result to verify the accuracy of the data. The findings of other models' evaluations are all taken from their original manuscripts. The primary reason with this is that the proposed technique reported in this article uses frameworks like vibrant word vectors and multichannel convolution to learn a wider range of interactional expression semantics, allowing it to identify more entity relations. When the number of channels increases, the recall rate does not increase significantly or even decreases. When the number of channels is too large, the model parameters increase, and the training time increases. To this end, this paper finally sets the number of multichannels to 4 and then conducts training and testing.

## 6. Conclusion

Biological entity relationship extraction is the basis for realizing intelligent medical care, which can improve the effect of intelligent medical question answering and promote the development of precision medical care. However, how to extract the relationship between biological entities from massive biomedical texts is a difficulty facing current life science experts and a hot spot in physical text mining. Therefore, this paper proposes a new multichannel convolution neural network model (MCCNN) for extracting the relationship between biological entities. The goal of this paper is to establish a universal system for removing various physical entity relationships, so only dynamic word embedding and position embedding information are input to the model so that the model can automatically extract the semantics of the expression relationship without manually designing features and the way to filter negative samples to improve the performance of the model. Through experimental comparison, it is shown that the method in this paper is effective on the task of biological entity relationship extraction. The following work plan is to use the trained model to mine massive biomedical literature, extract structured biological entity relationships, and establish an open-source database for life science researchers to use.

## Figures and Tables

**Figure 1:** Biological entities interact during cellular metabolism.

**Figure 2:** Compound-protein relationship extraction.

**Figure 3:** Overview of the method.

**Figure 4:** Structure of the multihead attention mechanism.

**Figure 5:** Performance of proposed work over different datasets.

**Figure 6:** Comparison over DDI dataset.

**Figure 7:** Comparison over CHEMPROT dataset.

**Figure 8:** Comparison of existing technique over both datasets.

**Table 1:** Dataset of biological entity interaction relationship.

Dataset	Entity type	Total	Positive sample	Negative samples	Positive and negative sample ratio
DDI [26]	Drug-drug	33 547	4 999	28 548	1 : 4.6
CHEMPROT [10]	Chemical protein	41 070	10 031	31 039	1 : 2.1

**Table 2:** Performance of proposed work over different datasets.

Dataset	Precision	Recall	F1-score
CHEMPROT	81.23	82.45	86.42
DDI	78.23	78.45	81.23

**Table 3:** Comparison over DDI dataset.

Approach	Precision	Recall	F1-score
SCNN	68.56	69.12	71.45
Joint AB-LSTM	75.85	77.21	78.51
MCCNN(proposed)	81.23	82.45	86.42

**Table 4:** Comparison over CHEMPROT dataset.

	Precision	Recall	F1-score
Transfer model	70.42	72.14	74.12
Ensemble model	64.1	65.14	68.45
GA-BGRU	71.24	75.21	79.12
MCCNN(proposed)	78.23	78.45	81.23

## Data Availability

The data shall be made available on request.
